RETRACTED

# Chemokine (C-C motif) ligand 18/membrane-associated 3/forkhead box O1 axis promotes the proliferation, migration, and invasion of intrahepatic cholangiocarcinoma

**DOI:** 10.1080/21655979.2022.2069383

**Published:** 2022-05-24

**Authors:** Chusi Wang, Hao Liang, Yanjie Li, Zhaofeng Tang, Yingcai Zhang

**Affiliations:** a Department of Hepatobiliary Surgery, The Third Affiliated Hospital, Sun Yat-sen University, Guangzhou, China; b Department of General Surgery, The Third Affiliated Hospital, Sun Yat-sen University, Guangzhou, China; c Department of Hepatic Surgery and Liver Transplantation Center of the Third Affiliated Hospital, Sun Yat-sen University, Guangzhou, China

**Keywords:** Phosphatidylinositol transfer protein, membrane-associated 3, chemokine (C-C motif) ligand 18, intrahepatic cholangiocarcinoma, forkhead box O1, nuclear factor kappa B

## Abstract

Phosphatidylinositol Transfer Protein, Membrane-Associated 3 (PITPNM3) often bind with chemokine (C-C motif) ligand 18 (CCL18) to promote tumor progression. However, the role of PITPNM3 in intrahepatic cholangiocarcinoma (ICC) is unclear. We first searched GEPIA database and detected the PITPNM3 expression using immunohistochemistry and real-time quantitative PCR. The results showed that PITPNM3 is high expression in ICC tissues and cells. Then we investigated the cell function of CLL18 and PITPNM3 through cell clone formation assay and transwell assay. The results indicated that CCL18 treatment promoted the proliferation, migration, and invasion of ICC cells. Silence of PITPNM3 reversed the effect of CCL18 on cell function. Simultaneously, we detected key protein expression of forkhead box O1 (FOXO1) and nuclear factor kappa B (NF-KB) through western blotting and found that CCL18 activated NF-KB pathway while inhibited FOXO1 pathway, the effect of which were attenuated by silence of PITPNM3. Finally, we confirmed which pathway affected the cell function using inhibitor of FOXO1 (AS1842856) and activator of NF-KB (Asatone). The results showed that AS1842856, not Asatone, relieved the inhibitory effect of si-PITPNM3 on the cell function of CCL18. In short, CCL18 treatment activated PITPNM3 to promote the proliferation, migration, and invasion of ICC via FOXO1 signaling pathway. These results provided a new insight for the diagnosis and therapy of ICC.

## Highlights

- PITPNM3 is high expression in ICC tissues and cells.
- Silence of PITPNM3 reversed the promotion effect of CCL18 on cell function.
- PITPNM3 promote ICC’ cell function via FOXO1 signaling pathway.

## Introduction

Intrahepatic cholangiocarcinoma (ICC), a kind of primary liver cancer, occurs proximal to the segmental biliary ducts and originates from the epithelial cells of the intrahepatic and extrahepatic bile ducts [1]. ICC is the second common primary liver cancer, the incidence of which is increasing in the whole world [2]. The outcome of patients with ICC is dismal owing to highly aggressive, lymph node metastasis, vascular invasion, late diagnosis, and lack of effective treatment options [2,3]. Therefore, further studies are needed to find the potential biomarkers at early stages and define the molecular mechanisms underlying ICC carcinogenesis.

RETRACTED

Phosphatidylinositol Transfer Protein, Membrane-Associated 3 (PITPNM3), also named PYK2 N-terminal domain interacting receptor 1, has been reported to have high expression in different cancers, such as oral squamous cell carcinoma [4], non-small cell lung cancer [5], and breast cancer [6]. Moreover, PITPNM3 often bind with chemokine (C-C motif) ligand 18 (CCL18) to promote tumor progression [4,6]. However, there is no report about PITPNM3 in ICC.

CCL18, belonging to beta-chemokine sub-family member, is produced by M2 tumor-associated macrophages (TAMs) to exert immunomodulatory functions [7–9]. Five receptors of CCL18 have been found, including G-protein coupled estrogen receptor, three types of C-C chemokine receptor (C-C Motif Chemokine Receptor 3, C-C Motif Chemokine Receptor 6, and C-C Motif Chemokine Receptor 8), and PITPNM3, in which PITPNM3 is believed to be the predominant receptor [7]. PITPNM3 receptor plays an important role in various malignancies by binding with CCL18 to stimulate calcium signaling [7]. However, the function of CCL18 is controversial. CCL18 plays the role of immunosuppression in non-small cell lung cancer, oral squamous cell carcinoma, and ovarian cancer; while plays the role of protection gastric cancer [4,5,10,11]. CCL18 affects tumor progression from two aspects. On the one hand, it directly acts on cancer cells by binding to PITPNM3 receptor [12]. On the other hand, it affects the progression of cancer cells by changing the tumor microenvironment [13]. Furthermore, CCL18 maybe a potential marker for diagnosis and a potential target of therapy [13]. However, the role of CCL18 in ICC is still unknown.

Therefore, we supposed that PITPNM3 participate in the progress of ICC, and CCL18 can activate PITPNM3. To validate our hypothesis, we first confirmed the expression and role of PITPNM3 on the proliferation, migration, and invasion of ICC tissues. Then we investigated whether CCL18 can activate PITPNM3 to regulate the development of ICC. Finally, we revealed the potential mechanism of CCL18 and PITPNM3 on the proliferation and metastasis of ICC. This study aims to confirm the role of PITPNM3 in ICC, and the goal is to provide new insight for the diagnosis and therapy of ICC and also provide a new clue for further study.

RETRACTED

## Materials and methods

### Gene expression profiling interactive analysis (GEPIA)

In our study, GEPIA database [14] (URL: http://gepia.cancer-pku.cn/detail.php?gene=PITPNM3) was used to evaluated the PITPNM3 expression in ICC. Additionally, the relationship between PITPNM3 expression and overall survival (or disease-free survival) was also determined in GEPIA database.

### Collection of patient tissue specimens

From 2014 to 2019, we collected 40 ICC tissues and paired paracancerous tissues at Third Affiliated Hospital of Sun Yat-sen University (China), from patients with ICC, who had surgery, to analyze the relationship between PITPNM3 expression and clinical parameters. Informed consents were obtained from all patients in our study by BioBank. Furthermore, our study was done according to the policies of the Institutional Research Ethics Committee of Third Affiliated Hospital of Sun Yat-sen University ([2019]02–177-01).

### Immunohistochemistry

The protein levels of PITPNM3 in ICC and paired paracancerous tissues were analyzed using immunohistochemistry (IHC) following a previous study with a few revisions [4,10]. Briefly, paraffin-embedded tissues were sliced into 5 μM section followed by dewaxing in xylene and rehydration in a graded alcohol series (100% ethanol, 90% ethanol, 70% ethanol, ddH_2_O). After that, the sections were heated for 15 min in citric acid buffer (pH 6.0) and then incubated with 3% H_2_O_2_ for 10 min, normal serum for 1 h at room temperature, anti-PITPNM3 primary antibody (1:500; #NBP2-34121; Novus, Littleton, CO, USA) overnight at 4°C, and HRP-Goat anti-rabbit IgG (1:500; #KS002; Jiancheng Bioengineering Institute, Nanjing, China) for 1 h at room temperature. Signals of PITPNM3 were visualized using DAB solution (#I025-1-1; Jiancheng Bioengineering Institute) following by counterstaining in hematoxylin for 15 s. Finally, the tissue sections were dehydrated in gradient ethanol and transparent in 100% xylene followed by sealing using neutral resin. The intensity of staining was scored as 0 (negative), 1 (weak), 2 (medium), and 3 (strong). The extent of IHC staining was based on the percentage of positive cells of positive tumor cells in the whole tissue slice. Intensity score and positive rate score were then multiplied to calculate the overall score. The protein expression was divided into low (score of 0–7) and high expression group (score of 8–12).

### Cell culture and cell treatment

Human Intrahepatic Biliary Epithelial Cells (HIBEC) was provided by Sciencell (San Diego, CA, USA) and was cultured in F-12 K (CellCook, Guangzhou, China) containing 10% fetal bovine serum (FBS, Gibco, Grand Island, NY, USA). QBC-939 was purchased from National Collection of Authenticated Cell Cultures and was kept in Roswell Park Memorial Institute (RPMI) 1640 culture medium supplementary with 10% FBS. HCCC-9810 cells were provided by CellCook and also kept in RPMI 1640 medium supplementary with 10% FBS. These three types of cells were amplified at an incubator supplemented with 5% CO_2_ at 37°C.

RETRACTED

For cell transfection, siRNA sequences, including siRNA-negative control (si-NC: CATCGCTGTGACGTTCTCTGTCCTT) and siRNA target for PITPNM3 (si-1: GAACTGTACCGGGTTTCCTTGAGAA, si-2: CATCTGCTCTGAGGCTTTCTCGCTT, si-3: CAGAGAGTTCCTGAAGTCCTCTGAT), were provided by Genepharma (Shanghai, China). Then they were transfected into HCCC-9810 cells using Lipofectamine 2000 reagent (Biosharp, Hefei, China) in accordance with the manufacturer’s instructions. The interference efficiency was further evaluated by real-time quantitative polymerase chain reaction (RT-qPCR) and western blotting at 48 h post-transfection.

For CCL18 (MedChemExpress, Shanghai, China), Asatone (MedChemExpress), and AS1842856 (MedChemExpress) treatment, HCCC-9810 cells were transfected with siRNAs for 24 h, then the final concentration of 10 μg/mL CCL18, 10 μM Asatone, or 100 nM AS1842856 was used to treat cells alone or simultaneously for another 48 h. After that, the cells were collected for further analysis.

### Western blotting

Western blotting was conducted following a previous study with few revisions [10]. The cells were lysed using RIPA (Beyotime, Shanghai, China) followed with protein quantification through BCA (Biosharp) method. Then 25 μg protein was used to electrophoresis on 10% sodium dodecyl sulfate and sodium salt polyacrylamide gel electrophoresis and transferred onto polyvinylidene fluoride (PVDF) membranes (Beyotime). After that, the membranes were blocked using 5% nonfat milk followed with washing thrice in Tris-buffered saline containing 0.1% Tween-20 (TBST). Then the membranes were incubated in the solution of following antibodies at 4°C overnight: PITPNM3 (Novus), p-P65 (ABCLONAL, Wuhan, China), P65 (Proteintech, Wuhan, China), p-FOXO1A (Abcam, Cambridge, MA, USA), FOXO1A (Abcam), and glyceraldehyde-3-phosphate dehydrogenase (GAPDH; Proteintech). After that, the membranes were washed with TBST for five times followed with incubation in peroxidase-conjugated secondary antibodies (Proteintech) for 1 h. The protein bands were visualized by enhanced chemiluminescence (Millipore, Temecula, USA). Image-Pro Plus 6.0 software (Thermo Fisher Scientific, Waltham, MA, USA) was used to get the gray value. After the target protein was normalized using GAPDH, we set the normalized value of si-NC group (Figure S2) or CCL18 group (Figure S4) as 1 to calculate the relative quantitative value of other groups.

RETRACTED

### RT-qPCR

RT-qPCR was conducted following a previous study with few revisions [10]. The cells were washed twice with phosphate-buffered saline (PBS) for three times. Total RNA was isolated from the cells using TriQuick Reagent (Solarbio, Beijing, China). Then total RNA (2 μg) was reversed to cDNA to follow the protocol of HiScript III RT SuperMix for qPCR (+gDNA wiper) (Vazyme, Nanjing, China). Finally, ChamQ Universal SYBR qPCR Master Mix (Vazyme) was used to perform qPCR on ABI 7500 system (Applied Biosystems, Foster city, CA, USA). The primers are as follows: PITPNM3 (forward: TTGGGATGAGCCAGTGGAAC; reverse: TGATGCTCGTCCAGTTTCCC) and GAPDH (forward: GAGTCAACGGATTTGGTCGT; reverse: GACAAGCTTCCCGTTCTCAG). The relative level of PITPNM3 was calculated normalized to GAPDH using 2^−ΔΔCt^.

### Cell clone formation assay

Cell clone formation assay was conducted following a previous study with few revisions [4]. The cells (500 cells per well) were seeded into the 6-well plate, and 5 mL per well medium containing 10% FBS was added into the plate. Then the cells were kept for 7 days. After that, the cells were fixed with 4% paraformaldehyde followed by staining in 1% crystal violet. The number of clones was counted as >50 cells/group.

### Transwell assay

Transwell assay was conducted following a previous study with few revisions [10]. HCCC-9810 cells were treated as indicated and then were collected and resuspended as the density of 2 × 10^6^ after digested using 0.25% trypsin. Thereafter, 24-well transwell plate (Corning, NY, USA) was used to perform Transwell assay according to standard protocol. In brief, for migration testing, a medium containing 10% FBS was added into the lower chamber, and 2 × 10^5^ HCCC-9810 cells in 100 μL RPMI 1640 with free FBS were added into the upper chamber. After incubation for 48 h at 37°C with 5% CO_2_, cotton swab was used to remove the cells that did not migrate through the inserts. The other cells that migrated to the underside of the insert were fixed in 4% paraformaldehyde and incubated for 15 min. After washing with PBS for two times, these cells were stained in 1% crystal violet for 10 min. The migrated cells were observed in inverted microscope followed by one-time washing with PBS. For invasion testing, little different from migration testing, the inserts were pre-coated with 100 μL of Matrigel mixture (dilution ratio: 1:5 in cold serum-free RPMI 1640) at an incubator with temperature 37°C and 5% CO_2_.

RETRACTED

### Statistical analysis

In our study, SPSS software (Standard version 16.0; IBM, Armonk, NY, USA) was used for the statistical analysis of data. The Student’s t test or analysis of variance was used to evaluate the difference of data from different groups. In addition, the correlation between PITPNM3 expression and the clinic-pathological characteristics were analyzed using Spearman rank correlation method. P value less than 0.05 was considered statistically significant.

## Results

Previous studies reported that PITPNM3 shows high expression in different cancers. Moreover, PITPNM3 acting as a predominant receptor plays an important role in various malignancies by binding with CCL18. Therefore, we supposed that PITPNM3 participates in the progress of ICC, and CCL18 can activate PITPNM3. To solve this problem, we first searched GEPIA database and detected the PITPNM3 expression using immunohistochemistry and real-time quantitative PCR. The results showed the PITPNM3 expression is high in ICC tissues and cells. Then we investigated the cell function of CLL18 and PITPNM3 through cell clone formation assay and transwell assay. The results indicated that CCL18 treatment promoted the proliferation, migration, and invasion of ICC cells. Silence of PITPNM3 reversed the effect of CCL18 on cell function. Simultaneously, we detected key protein expression of FOXO1 and NF-KB through western blotting and found that CCL18 activated NF-KB pathway while inhibited FOXO1 pathway, the effects of which were attenuated by silence of PITPNM3. Finally, we confirmed which pathway affects the cell function using inhibitor of FOXO1 (AS1842856) and activator of NF-KB (Asatone), The results showed that AS1842856, not Asatone, relieved the inhibitory effect of si-PITPNM3 on the cell function of CCL18.

### PITPNM3 is high expression in ICC tissues

To investigate the PITPNM3 expression in ICC, we first search GEPIA database. The results showed that PITPNM3 shows overexpression in ICC tissues compared to paracancerous tissues (Figure 1(a)). Moreover, high expression of PITPNM3 had lower overall survival (P = 0.48) and disease-free survival (P = 0.28) than those with low expression of PITPNM3 in ICC tissues (Figure 1(b)). These results indicated that high expression of PITPNM3 maybe having poor prognosis. To further confirm the above findings, we collected 40 ICC tissues and paired paracancerous tissues to test PITPNM3 expression via IHC. The results showed that PITPNM3 expression was elevated in ICC tissues compared to paired paracancerous tissues (Figure 1(c)). Additionally, we found that high expression of PITPNM3 was closely related to poor overall survival (P = 0.005) and disease-free survival (P = 0.003) in ICC (Figure 1(d)). In detail, the clinicopathologic characteristics of tumor size and lymph node metastasis had significant difference between the high expression of PITPNM3 (N = 22) and low expression of PITPNM3 (N = 18) in ICC tissues (Table 1). The above results suggested that PITPNM3 shows high expression in ICC tissues, which is related with poor prognosis.

RETRACTED

**Table 1.** Relationship between PITPNM3 expression and clinicopathological parameters

Variable	High expression of PITPNM3	Low expression of PITPNM3	*P* value
Age (year)			0.869
≤55	8	7	
>55	14	11	
Pathologic subtype			0.229
Well	1	3	
Moderately poorly	13 8	12 3	
Gender			0.603
Male	14	10	
Female	8	8	
CA-199 (U/mL)			0.679
≤35	3	4	
>35 Tumor number single multiple Tumor size (cm) ≤5 >5 Vascular invasion yes no	19 18 4 6 16 12 10	14 17 1 11 7 6 12	0.355 0.031* 0.215
T stage			0.660
T1(1a&1b)	9	9	
T2 T3(3a&3b)	10 3	8 1	
N stage			0.035*
Negative	12	16	
Positive	10	2	
TNM stage (AJCC) ^a^			0.083
I(IA&IB)	5	10	
II III(IIIA&IIIB)	6 11	4 4	

*:Chi-square(and Fisher’s exact) test, P value<0.05.

a: American Joint Committee on Cancer (AJCC); patients were staged in accordance with the 8th Edition of the AJCC Cancer’s TNM Classification.

**Figure 1.** PITPNM3 shows high expression and corrected with poor prognosis in intrahepatic cholangiocarcinoma tissues. (a) GEPIA (gene expression profiling interactive analysis) database showed that PITPNM3 is overexpressed in intrahepatic cholangiocarcinoma tissues compared to paracancerous tissues. (b) GEPIA database showed that high expression of PITPNM3 had lower overall survival and disease-free survival than those with low expression of PITPNM3 in intrahepatic cholangiocarcinoma tissues. (c) Immunohistochemistry was used to test PITPNM3 expression in intrahepatic cholangiocarcinoma tissues and paired paracancerous, N = 40. (d) High expression of PITPNM3 was closely related to poor survival and disease-free survival in intrahepatic cholangiocarcinoma.

### PITPNM3 is overexpressed in ICC cells, and its expression was inhibited efficiently by siRNAs target for PITPNM3

To further investigate the PITPNM3 expression in ICC cells, we collected ICC cells (including QBC-939 and HCCC-9810) and HIBEC (as control cells). RT-qPCR results showed that PITPNM3 expression was upregulated about 5-fold in QBC-939 cells and about 7-fold in HCCC-9810 cells when compared to those in HIBEC (Figure 2(a)). Western blotting results also showed that PITPNM3 expression climed up in QBC-939 (about 2-fold) and HCCC-9810 (about 3-fold) cell lines compared to HIBEC cells (Figure 2(b,c)). These results also confirmed that the expression of PITPNM3 is high in ICC cells, and HCCC-9810 cells had the highest expression of PITPNM3. Therefore, we selected HCCC-9810 cells for further study. We first synthesized siRNAs target for PITPNM3 and then transfected into cells for 48 h. RT-qPCR results showed that all siRNAs (including si-1, si-2, si-3) interfere with the PITPNM3 expression in HCCC-9810 cells compared to the si-NC group, in which si-1 and si-2 decreased about 2-fold and si-3 decreased about 5-fold (Figure 2(d)). Therefore, we selected cells in si-NC and si-3 groups to perform western blotting validation, and the results showed that si-3 significantly reduced PITPNM3 expression (about 3-fold) in HCCC-9810 cells than in si-NC group (Figure 2(e,f)). These results indicated that PITPNM3 expression can be silenced efficiently by si-3. In short, the above results suggested that PITPNM3 is overexpressed in ICC cells, and si-3 can efficiently inhibit PITPNM3 expression in HCCC-9810 cells.

RETRACTED

**Figure 2.** PITPNM3 is overexpressed in intrahepatic cholangiocarcinoma cells, and its expression was inhibited efficiently by siRNAs target for PITPNM3. (a) Real-time quantitative polymerase chain reaction was used to evaluate PITPNM3 (membrane-associated 3) expression in QBC-939 and HCCC-9810 cells and control cells HIBEC. (b, c) Western blotting was used to detect PITPNM3 expression in QBC-939 and HCCC-9810 cells and control cells HIBEC. (d) Real-time quantitative polymerase chain reaction was used to assess the interference efficiency of siRNAs target for PITPNM3 in HCCC-9810 cells. si-NC is the siRNA negative control, and si-1, si-2, and si-3 are the siRNA sequence target for PITPNM3. (e, f) Western blotting was used to determine the PITPNM3 expression in HCCC-9810 cells after si-NC and si-3 transfected for 48 h.

### Silence of PITPNM3 reversed the promotion effect of CCL18 on proliferation, migration, and invasion of HCCC-9810 cells

Then we investigate the function of PITPNM3 in ICC. Previous study showed that PITPNM3 is a receptor of CCL18 [7]. So, we treated cells using 10 μg/mL CCL18 after si-NC or si-3 was transfected into HCCC-9810. Then the ability of cell proliferation, migration, and invasion was evaluated via cell clone formation assay and transwell assay. The results showed that relative to si-NC group, silence PITPNM3 obviously decreased the ability of cell proliferation, migration, and invasion, and CCL18 significantly promoted the ability of cell proliferation, migration, and invasion (Figure 3(a–c)). Moreover, interference of the PITPNM3 expression reversed the effects of CCL18 on cell function (Figure 3(a–c)). The above results suggested that silence of PITPNM3 reversed the promotion effect of CCL18 on proliferation, migration, and invasion of HCCC-9810 cells.

RETRACTED

**Figure 3.** Silence of PITPNM3 reversed the promotion effect of CCL18 on proliferation, migration, and invasion of HCCC-9810 cells. si-NC or si-3 was first transfected into HCCC-9810 cells for 24 h then were treated by 10 μg/mL CCL18 for 48 h, then cell clone formation assay and Transwell assay were used to evaluate the proliferation (a), migration (b), and invasion (c). PITPNM3: membrane-associated 3; CCL18: chemokine (C-C motif) ligand 18; si-NC is the siRNA negative control, si-3 is the siRNA sequence target for PITPNM3.

### Knockdown of PITPNM3 expression attenuates the activation effect of CCL18 on NF-kappa B and its inhibitory effect on FOXO1 signaling

Next, we explored the potential mechanism. Previous studies reported that CCL18 can activate the NF-kB signaling pathway [15]. In addition, Forkhead box protein O1 (FOXO1) is a regulator of TAMs that secrete anti-inflammatory cytokines and chemokines [16,17]. Therefore, we conducted western blotting to evaluate p-P65 and p-FOXO1A expression. The results showed that relative to si-NC group, knockdown of PITPNM3 expression obviously decreased the p-P65 expression and increased p-FOXO1A expression; CCL18 treatment promoted the expression of p-P65 while inhibited p-FOXO1A expression compared to si-NC group, and knockdown of PITPNM3 attenuated the effect of CCL18 on the expression of p-P65 and p-FOXO1A (Figure 4(a–e)). In conclusion, silence of PITPNM3 expression attenuates the activation effect of CCL18 on NF-kappa B and its inhibitory effect on FOXO1 signaling.

**Figure 4.** Knockdown of PITPNM3 expression attenuates the activation effect of CCL18 on NF-kappa B and its inhibitory effect on FOXO1 signaling. (a) Western blotting was used to evaluate the expression of p-P65, P65, p-FOXO1A, and FOXO1A. (b-e) Protein quantification of bands in A picture was performed using Image-Pro Plus 6.0 software. PITPNM3: membrane-associated 3; CCL18: chemokine (C-C motif) ligand 18; forkhead box O1.

### CCL18 regulate the cell function in HCC-9810 cells via PITPNM3/FOXO1 signaling pathway

To further confirm whether NF-kB and FOXO1 signaling pathway participate in CCL18/PITPNM3 axis regulating the function of ICC cells, we treated HCCC-9810 cells using the activator of NF-kB (Asatone) or FOXO1 inhibitor (AS1842856) combined with CCL18. We found that interference of PITPNM3 inhibited the promotion effect of CCL18 on proliferation, migration, and invasion of HCCC-9810 cells, and these results are the same as Figure 3(a–c); however, these inhibition effects were relieved by AS1842856 but not Asatone (Figure 5(a–c)). The above results indicated that CCL18 maybe regulate the proliferation, migration, and invasion via PITPNM3/FOXO1 signaling pathway.

RETRACTED

**Figure 5.** CCL18 regulate the cell function in HCC-9810 cells via PITPNM3/FOXO1 signaling pathway. si-NC or si-3 was transfected into HCCC-9810 cells for 24 h and then were treated by 10 μg/mL CCL18 with or without 10 μM Asatone (or 100 nM As1842856) simultaneously for 48 h, then cell clone formation assay and Transwell assay were used to evaluated the proliferation (a), migration (b), and invasion (c). PITPNM3: membrane-associated 3; CCL18: chemokine (C-C motif) ligand 18; forkhead box O1.

## Discussion

ICC is a rare but devastating malignancy with late onset and presents a high mortality if there is no treatment, and complete extirpation of the tumor (including R0 resection, which can be detected under microscope) is the best possibility for long-term survival of patients with ICC [18]. Therefore, it is a major oncological challenge to optimally diagnose, stage, and manage ICC, which need more studies to solve [19]. PITPNM3 and CCL18 are reported to participate in cancer cell activation, migration, and the progress of immune tolerance [20,21]. In this study, we also found that PITPNM3 shows high expression in ICC tissues and cells. CCL18 treatment promoted the proliferation, migration, and invasion of ICC cells. Silence of PITPNM3 reversed the effect of CCL18 on cell function. Simultaneously, CCL18 activated NF-KB pathway while inhibited FOXO1 pathway, effects of which were attenuated by silence of PITPNM3. Furthermore, AS1842856, not Asatone, relieved the inhibitory effect of si-PITPNM3 on the cell function of CCL18.

PITPNM3, one of member of a large family of G protein-coupled receptors, promotes the development of different cancer, such as in hepatic carcinoma, mitofusin-2 could interact with transcription factor SP1 to suppress PITPNM3 expression, which contributed to the inhibition of tumor [21]. Therefore, PITPNM3 can be a target for therapy, for instance, pachymic acid, a lanostrane-type triterpenoid from P.cocos., suppressed breast cancer metastasis via inhibiting PITPNM3 expression [12]. In our study, we revealed that PITPNM3 expresses high expression in ICC tissues and cells, and silence of PITPNM3 reduces ICC cells proliferation, migration, and invasion.

Previous study showed that PITPNM3 is a receptor of CCL18 [7]. CCL18 is mainly produced by M2 tumor-associated macrophages [8]. The role of CCL18 is controversial. Leung SY et al. reported that high expression of CCL18 prolonged the overall survival time of patients with gastric cancer [11]. However, in most kind of cancers, CCL18 acted as a promoter. For example, CCL18 stimulation promoted the migration and invasion of breast cancer cells, which was induced by PCAF-dependent acetylation [22]. The CCL18 promoted the development of ovarian cancer through mTORC2 pathway and proline-rich tyrosine kinase 2 signaling pathway [23,24]. In addition, the promotion effect of CCL18 on oral squamous cell carcinoma cell proliferation and metastasis by inducing linc00319 expression to regulate miR-199a-5p/frizzled class receptor 4 axis [25]. Moreover, for oral squamous cell carcinoma, CCL18 level is an independent prognostic factor of overall and disease-free survival time [26]. For colorectal cancer, CCL18 expression level is also an independent favorable prognostic biomarker [27]. For human pancreatic ductal adenocarcinoma (PDAC), serum CCL18 is a potential biomarker of diagnosis and prognosis and have been found promoting the epithelial–mesenchymal transition (EMT), invasion, and migration of pancreatic cancer cells [28]. Similar to most types of cancers, we confirmed that CCL18 stimulation increased the ICC cells proliferation and metastasis.

RETRACTED

In addition, CCL18 can bind with PITPNM3, inducing EMT, migration, and invasion of non-small cell lung cancer and breast cancer via PI3K/Akt/GSK3β/Snail signaling pathway and engulfment and cell motility 1/dedicator of cytokinesis protein 4 CRK binding protein signaling pathway, respectively [5,6]. CCL18/PITPNM3 axis also activates JAK2/STAT3 signaling pathway to promote the growth and metastasis of oral squamous cell carcinoma cells [4]. Furthermore, CCL18/NF-kB/vascular cell adhesion molecule 1 pathway was activated by tumor-associated macrophages, which promotes progression of PDAC [29]. Additionally, previous study showed that CCL18/PITPNM3 activated NF-kB signaling to enhance migration, invasion, and EMT of liver cancer cells [15]. Therefore, we detected whether CCL18 treatment can activate PITPNM3 to regulate NF-kB signaling pathway in ICC. The results showed that CCL18 activated NF-kB signaling pathway, and interference of PITPNM3 reduced this effect. However, the activator of NF-kB signaling pathway Asatone had no effect on ICC proliferation and metastasis. Maybe the CCL18 treatment can be activated NF-kB signaling pathway; however, there are other factors that affect the ICC proliferation and metastasis.

FOXO1, a member of the forkhead box O family of transcription factors, has been reported as a regulator of TAMs [16]. Previous literature reported that TAMs can secrete anti-inflammatory cytokines and chemokines, including arginase 1, CCL18, and C-C motif chemokine ligand 20 [17]. The effect of FOXO1 in different cancers is also controversial. For breast cancer [30], bladder cancer [31], and cervical cancer [32], FOXO1 deficiency indicates worse clinical outcomes through inducing cell cycle arrest and apoptosis [33]. However, for urothelial carcinoma, FOXO1 amplification indicates poor prognosis [34]. Therefore, we also detected whether FOXO1 pathway involved in CCL18/PITPNM3 mediated the cell function in ICC. The results presented that CCL18 inhibited the activity of FOXO1 and promoted cell proliferation, migration, and invasion. However, silence of PITPNM3 reversed the effect of CCL18 on the activity of FOXO1 and cell function. Furthermore, inhibitor of FOXO1 signaling pathway, AS1842856, rescues the ability of proliferation, migration, and invasion in si-PITPNM3+ CCL18 cells. These results indicated that inhibition of FOXO1 may contribute to the development of ICC, and CCL18/PITPNM3 axis can promote the proliferation, migration, and invasion of ICC by regulating FOXO1 signaling pathway.

RETRACTED

However, our study on in vivo experiment to validate CCL18/PITPNM3 axis can promote the progression of ICC by regulating FOXO1 signaling pathway. Moreover, the expression of CCL18 and PITPNM3 in ICC patients also need further study. Thereby, we will collect more tissue samples and serum samples from ICC patient to confirm the expression of CCL18 and PITPNM3 and further analyse the relationship between their expression and clinicopathologic characteristics. Additionally, we will add in vivo experiment to further confirm our conclusion.

## Conclusion

Taken together, PITPNM3 is overexpressed in ICC tissues and cells. Moreover, CCL18 activated PITPNM3 to promote the proliferation, migration, and invasion of ICC by regulating FOXO1 signaling pathway. These results provided a new insight for the diagnosis and therapy of ICC and also provided new clues for further study.
